The article "Introduction and Utilization of High Priced HCV Medicines across Europe; Implications for the Future" was published in 2016. Journal: Front Pharmacol.

# Introduction and Utilization of High Priced HCV Medicines across Europe; Implications for the Future

**DOI:** 10.3389/fphar.2016.00197

**Published:** 2016-07-22

**Authors:** Winnie de Bruijn, Cristina Ibáñez, Pia Frisk, Hanne Bak Pedersen, Ali Alkan, Patricia Vella Bonanno, Ljiljana S. Brkičić, Anna Bucsics, Guillaume Dedet, Jaran Eriksen, Joseph O. Fadare, Jurij Fürst, Gisselle Gallego, Isabella P. Godói, Augusto A. Guerra Júnior, Hakkı Gürsöz, Saira Jan, Jan Jones, Roberta Joppi, Saim Kerman, Ott Laius, Newman Madzikwa, Einar Magnússon, Mojca Maticic, Vanda Markovic-Pekovic, Amos Massele, Olayinka Ogunleye, Aisling O'Leary, Jutta Piessnegger, Catherine Sermet, Steven Simoens, Celda Tiroyakgosi, Ilse Truter, Magnus Thyberg, Kristina Tomekova, Magdalena Wladysiuk, Sotiris Vandoros, Elif H. Vural, Corinne Zara, Brian Godman

**Affiliations:** ^1^Department of Pharmaceutical Sciences, Utrecht UniversityUtrecht, Netherlands; ^2^Catalan Health Service - Servei Català de la SalutBarcelona, Spain; ^3^Public Health Services Committee, Stockholm County CouncilStockholm, Sweden; ^4^Health Technologies and Pharmaceuticals, Division of Health Systems and Public Health, WHO Regional Office for EuropeCopenhagen, Denmark; ^5^Turkish Medicines and Medical Devices Agency, Ministry of HealthAnkara, Turkey; ^6^Independent Pharmaceutical ConsultantMellieha, Malta; ^7^Croatian Health Insurance FundZagreb, Croatia; ^8^Department of Finance, University of ViennaVienna, Austria; ^9^Ministry of HealthParis, France; ^10^Division of Clinical Pharmacology, Department of Laboratory Medicine, Karolinska Institutet, Karolinska University Hospital HuddingeStockholm, Sweden; ^11^Department of Pharmacology, Ekiti State UniversityAdo-Ekiti, Nigeria; ^12^Health Insurance InstituteLjubljana, Slovenia; ^13^School of Medicine, The University of Notre Dame AustraliaDarlinghurst, NSW, Australia; ^14^Department of Pharmacology and Clinical Neuroscience, Umea UniversityUmea, Sweden; ^15^School of Pharmacy, Graduate Program in Medicines and Pharmaceutical Assistance, Federal University of Minas GeraisBelo Horizonte, Brazil; ^16^Department of Social Pharmacy, SUS Collaborating Centre – Health Technology Assessment and Excellence in Health, College of Pharmacy, Federal University of Minas GeraisBelo Horizonte, Brazil; ^17^Clinical Pharmacy, Rutgers State University of New JerseyPiscataway, NJ, USA; ^18^Horizon Blue Cross Blue Shield of New JerseyNewark, NJ, USA; ^19^Scottish Medicines ConsortiumGlasgow, UK; ^20^Pharmaceutical Drug Department, Azienda Sanitaria Locale of VeronaVerona, Italy; ^21^State Agency of MedicinesTartu, Estonia; ^22^Ministry of Health and Child CareHarrare, Zimbabwe; ^23^Department of Health Services, Ministry of HealthReykjavík, Iceland; ^24^Clinic for Infectious Diseases and Febrile Illnesses, University Medical Centre LjubljanaLjubljana, Slovenia; ^25^Faculty of Medicine, University of Banja LukaBanja Luka, Bosnia and Herzegovina; ^26^Ministry of Health and Social WelfareBanja Luka, Bosnia and Herzegovina; ^27^Department of Clinical Pharmacology, School of Medicine, University of BotswanaGaborone, Botswana; ^28^Clinical Pharmacology Unit, Department of Medicine, Lagos State University Teaching HospitalLagos, Nigeria; ^29^Department of Pharmacology and Therapeutics, Lagos State University College of MedicineLagos, Nigeria; ^30^National Centre for PharmacoeconomicsDublin, Ireland; ^31^Hauptverband der Österreichischen SozialversicherungsträgerWien, Austria; ^32^IRDESParis, France; ^33^Department of Pharmaceutical and Pharmacological Sciences, KU LeuvenLeuven, Belgium; ^34^Ministry of Health, Nelson Mandela DriveGaborone, Botswana; ^35^Drug Utilisation Research Unit, Faculty of Health Sciences, Nelson Mandela Metropolitan UniversityPort Elizabeth, South Africa; ^36^Stockholms Läns Landsting, Hälso-och SjukvårdsförvaltningenStockholm, Sweden; ^37^Faculty of Management, Comenius UniversityBratislava, Slovakia; ^38^HTA ConsultingCracow, Poland; ^39^School of Management and Business, King's College LondonLondon, UK; ^40^Strathclyde Institute of Pharmacy and Biomedical Sciences, University of StrathclydeGlasgow, UK

**Keywords:** boceprevir, cross national drug utilization study, demand-side measures, Hepatitis C, introduction new medicines, sofosbuvir, telaprevir

The article "Introduction and Utilization of High Priced HCV Medicines across Europe; Implications for the Future" was published in 2016. Journal: Front Pharmacol.

## Abstract

**Background:** Infection with the Hepatitis C Virus (HCV) is a widespread transmittable disease with a diagnosed prevalence of 2.0%. Fortunately, it is now curable in most patients. Sales of medicines to treat HCV infection grew 2.7% per year between 2004 and 2011, enhanced by the launch of the protease inhibitors (PIs) boceprevir (BCV) and telaprevir (TVR) in addition to ribavirin and pegylated interferon (pegIFN). Costs will continue to rise with new treatments including sofosbuvir, which now include interferon free regimens.

**Objective:** Assess the uptake of BCV and TVR across Europe from a health authority perspective to offer future guidance on dealing with new high cost medicines.

**Methods:** Cross-sectional descriptive study of medicines to treat HCV (pegIFN, ribavirin, BCV and TVR) among European countries from 2008 to 2013. Utilization measured in defined daily doses (DDDs)/1000 patients/quarter (DIQs) and expenditure in Euros/DDD. Health authority activities to influence treatments categorized using the 4E methodology (Education, Engineering, Economics and Enforcement).

The article "Introduction and Utilization of High Priced HCV Medicines across Europe; Implications for the Future" was published in 2016. Journal: Front Pharmacol.

**Results:** Similar uptake of BCV and TVR among European countries and regions, ranging from 0.5 DIQ in Denmark, Netherlands and Slovenia to 1.5 DIQ in Tayside and Catalonia in 2013. However, different utilization of the new PIs vs. ribavirin indicates differences in dual vs. triple therapy, which is down to factors including physician preference and genotypes. Reimbursed prices for BCV and TVR were comparable across countries.

**Conclusion:** There was reasonable consistency in the utilization of BCV and TVR among European countries in comparison with other high priced medicines. This may reflect the social demand to limit the transmission of HCV. However, the situation is changing with new curative medicines for HCV genotype 1 (GT1) with potentially an appreciable budget impact. These concerns have resulted in different prices across countries, with their impact on budgets and patient outcomes monitored in the future to provide additional guidance.

## Introduction

The incidence and prevalence of patients with hepatitis C virus (HCV) infection is growing. However, the true worldwide incidence remains unknown due to heterogeneous registration and case definitions (European Centre for Desease Prevention Control, 2010). Overall, it is believed that the diagnosed global prevalence of HCV is approximately 2.0% (1.7–2.3%) for adults, which corresponds to approximately 104 (87–124) million persons world-wide (Table 1; McGowan et al., 2013; Mohd Hanafiah et al., 2013; European Association for the Study of the Liver, 2014; Hope et al., 2014; Wedemeyer et al., 2015). Others have suggested higher figures at 2.8% globally (Lemoine and Asia, 2014), leading to estimated prevalence rates of 150–184 million world-wide (Ramachandran et al., 2012; Mohd Hanafiah et al., 2013; Lemoine and Asia, 2014; Phelan and Cook, 2014; Barua et al., 2015; Cure et al., 2015; Norton, 2015; Fraser et al., 2016), with approximately 85% of patients living in low to middle income (LMIC) countries (Phelan and Cook, 2014). However, estimated figures for South Africa are lower at 0.1–1.7% (Fraser et al., 2016). In 2013, diagnosis rates vs. the estimated prevalence rates varied from 81% in Sweden and 43% in Belgium to just 16% in Turkey (Table 1; Dore et al., 2014; Wedemeyer et al., 2015).

**Table 1:** **Reported anti-HCV prevalence rates (adjusted for the adult population), genotype 1 (GT1) distribution and estimated diagnose and treatment rate (Dore et al., 2014; Gower et al., 2014; Hope et al., 2014; Wedemeyer et al., 2015)**.

	**AU**	**BE**	**DK**	**EE**	**ES**	**FR**	**HR**	**IT**	**NL**	**SE**	**TR**	**UK**
Adult anti-HCV	0.5%	0.9%	0.7%	–	1.7%	0.6%	–	2.0%	0.2%	0.7%	1.0%	0.6%
prevalence	(0.1–0.7%)	(0.1–1.2%)	(0.5–0.7%)		(0.4–2.6%)	(0.4–1.1%)		(1.6–7.3%)	(0.1–0.4%)	(0.5–0.7%)	(0.6–2.1%)	(0.4–1.2%)
Genotype 1a	20.3%	–	34.0%	1.0%	25.5%	14.8%	13.1%	4.2%	14.8%	38.2%	8.1%	24.4%
Genotype 1b	51.6%	50.4%	12.0%	71.0%	43.8%	29.7%	37.4%	57.5%	15.7%	7.0%	83.7%	11.9%
Genotype 1c	–	8.6%	–	–	–	–	–	–	–	–	–	–
Estimated diagnosed rate (2013)	37%	43%	59%	–	40%	69%	–	–	61%	81%	16%	35%

NB: AU, Austria; BE, Belgium; DK, Denmark; EE, Estonia; ES, Spain; FR, France; HR, Croatia; IT, Italy; NL, the Netherlands; SE, Sweden; TR, Turkey; UK, United Kingdom.

The article "Introduction and Utilization of High Priced HCV Medicines across Europe; Implications for the Future" was published in 2016. Journal: Front Pharmacol.

Annually up to 0.5 million people die from the consequences of chronic hepatitis C infection, mainly in Africa, Asia and Eastern Europe (Lozano et al., 2012). Most people are unaware of their HCV infection due to the slow progress of the disease (Yehia et al., 2014), with sequelae of chronic hepatitis potentially appearing up to 20–30 years later. These include liver cirrhosis, which occurs in 10–20% of patients with hepatitis C, and develops into a 1–5% annual risk of hepatocellular carcinoma and 3–6% annual risk of hepatic decompensation (Thein et al., 2008; Westbrook and Dusheiko, 2014). In 2012, cirrhosis of the liver was the tenth leading cause of death in LMIC countries (globally the twelfth leading cause), with liver cancer the ninth leading cause of death in upper-middle-income countries (globally the sixteenth leading cause) (World Health Organisation, 2012; Lemoine and Asia, 2014).

Until 2011, treatment choices and their effectiveness were limited, especially for patients with genotype 1 (GT1). GT1 HCV-patients account for up to 60% of HCV infections worldwide, and predominate in Eastern, Northern and Southern Europe as well as North America and Japan (Schalm et al., 1997; McHutchison et al., 1998; Poynard et al., 1998; Cebolla and Björnberg, 2012; Messina et al., 2014). Cure rates, defined as sustained virological response (SVR), were typically only seen in 35–43% of patients with GT1 following dual therapy with ribavirin and pegylated interferons (pegIFNs) (Schalm et al., 1997; McHutchison et al., 1998; Poynard et al., 1998; Manns et al., 2013; Mathurin, 2013; Chou et al., 2014; Kohli et al., 2014). However, the serious side-effects associated with these treatments, coupled with complex regimens, resulted in problems with adherence. This led to less than 50% of patients typically completing their treatment course (McHutchison et al., 2002; Lo Re et al., 2011; Brennan and Shrank, 2014).

In 2011, the direct acting antivirals (DAAs) boceprevir (BCV), and telaprevir (TVR) became available (Chou et al., 2014)^1^^,^^2^. BCV and TVR are only licensed for GT1. Consequently physicians need to test for genotypes before starting treatment^1, 2^. BCV and TVR improved SVR (RR, 2.05; 95% CI 1.70–2.48) when combined with ribavirin and pegIFNs (triple therapy) (Chou et al., 2014; Kohli et al., 2014; Manzano-Robleda et al., 2015)^3^; however, there were more adverse events (RR, 1.05; 1–1.03; NNH 77.59) (Manzano-Robleda et al., 2015). In recent years, second generation DAAs have become available with encouraging cure rates up to 90–95% of patients, potentially providing shorter treatment courses and less side effects than previous treatment approaches (Kohli et al., 2014; Childs-Kean and Hand, 2015)^3^. These were sofosbuvir, simeprevir, daclatasvir and ledipasvir approved by the European Medicine Agency (EMA) in late 2013 and 2014^4^^,^^5^^,^^6^^,^^7^. More recently, combinations of DAAs have also been approved by EMA providing further options for highly effective, safe and well tolerated treatment of HCV GT1 patients (Kohli et al., 2014)^8^.

The article "Introduction and Utilization of High Priced HCV Medicines across Europe; Implications for the Future" was published in 2016. Journal: Front Pharmacol.

These developments resulted in the anti HCV therapeutics market expanding at a compounded annual growth rate (CAGR) of 2.7% between 2004 and 2011^9^^,^^10^, with growth rates appreciably higher after this^10^. This has resulted in worldwide sales of sofosbuvir already at US$12.4 billion in 2014 (Trooskin et al., 2015). In the US, treatments for hepatitis C became the fourth most expensive speciality medicine class in 2014 with sofosbuvir already capturing 37.5% of the HCV market^11^. These growth rates in expenditure are due not only to the price of these new treatments at over US$50,000/patient/course in some countries, but also the effectiveness and limited side-effects of the second generation DAAs (Mohd Hanafiah et al., 2013; Brennan and Shrank, 2014; Senior, 2014). In addition, these new treatments are being used in patients with advanced liver disease, such as those with decompensated cirrhosis awaiting transplantation, appreciably increasing the pool of eligible patients.

We are already seeing that some European health authorities are unable to fund new high priced medicines, exacerbated by their continual launch (Experts in Chronic Myeloid Leukemia, 2013; Kantarjian et al., 2013; Godman et al., 2015)^12^. This will impact on available funding for new treatments for HCV despite their undoubted effectiveness (Brennan and Shrank, 2014; Lemoine and Asia, 2014; Trooskin et al., 2015; Norton, 2015). The arrival of cost-effective second generation DAAs has fuelled the debate over pricing and reimbursement decisions across Europe given typically reimbursement for new expensive cancer treatments and those for orphan diseases despite often limited health gain, as well as whether there should be a greater focus on the budget impact of new medicines rather than just their cost-effectiveness (Kantarjian et al., 2013; Simoens et al., 2013; Cohen and Felix, 2014; Godman et al., 2015; Messori, 2015a)^13^.

The article "Introduction and Utilization of High Priced HCV Medicines across Europe; Implications for the Future" was published in 2016. Journal: Front Pharmacol.

Consequently, the aim of this initial study is to compare the uptake of BCV and TVR among European countries from a health authority perspective alongside implemented activities to influence their prescribing. We will subsequently build on the findings, including current activities among health authorities regarding second generation DAAs including price negotiations, to provide future direction and guidance to health authorities (Civaner, 2012; Lemoine and Asia, 2014)^10^. This will involve specific studies to ascertain utilization and expenditure of second generation DAAs alongside negotiated prices.

## Methods

This was a retrospective cross sectional descriptive observational study involving twelve countries and regions from across Europe. Health authorities were contacted to provide aggregated data on the utilization and expenditure of BCV and TVR. This was purely voluntary as there was no funding for them and no funding to purchase utilization data from commercial sources. We have used this approach before when analysing the influence of different health authority measures to enhance the prescribing of generic atypical antipsychotics, proton-pump inhibitors, renin-angiotensin inhibitors, selective serotonin re-uptake inhibitors and statins across Europe (Godman et al., 2010a, 2014a; Vonèina et al., 2011; Moon et al., 2014).

The European countries and regions that provided utilization and expenditure data typically cover 100% of their population. However, there are differences in their geography, i.e., central, eastern, and western European countries, epidemiology, and financing of as well as available resources for healthcare (Table 2). This is important given the heterogeneity of European healthcare systems and suggested approaches when conducting cross national studies (Cacace et al., 2013). The only exception to health authority data is Turkey, where data from the Ministry of Health were sourced from Intercontinental Marketing Services (IMS).

**Table 2:** **Details of methods of financing healthcare, GDP spent on health and data providers (Godman et al., 2010a, 2013a; Atun et al., 2013; Hesse et al., 2013)^14^**.

**Country/region**	**Taxation/health insurance**	**GDP/capita (PPP in US $)**	**% GDP spent on health (2010–2014)**	**Data providers (100% coverage of population unless otherwise stated)**
Austria (AT)	Health Insurance	43,390	11.0	Data Warehouse of the Federation of Austrian Social Insurance Institutions—covers 98% of the population
Belgium (BE)	Health Insurance	39,860	11.2	National Institute for Health and Disability Insurance (INAMI-RIZIV)
Croatia (HR)	Health Insurance	18,760	7.3	Croatian Health Insurance Fund covering over 99% of the population. HCV treatments funded from a separate budget for expensive medicines
Denmark (DK)	Taxation	43,430	10.6	Danish Prescription Registry
Estonia (EE)	Health Insurance	22,500	5.7	Estonian Health Insurance Fund
France	Health Insurance	38,847	11.8	SNIIRAM (The National Information System of public Health Insurances)
Italy (IT)	Taxation	32,920	9.1	Medicines Utilization Unit's elaboration of data from Osmed Database and Tracciabilità del farmaco
The Netherlands (NL)	Health Insurance	43,510	12.9	The Drug Information System of Dutch National Health Care Institute
Slovenia (SI)	Health Insurance	27,240	9.2	The National Institute of Public Health and Health Insurance Institute Prescription database
Spain—Catalonia (ES—CT)	Taxation	31,670	8.9	Catalan Health Service drug prescription database (DATAMART)
Sweden (SE)	Taxation	43,980	9.7	National Swedish Prescribed Drug Register
Turkey (TR)	Health Insurance	18,020	5.6	Utilization information from the Ministry of Health sourced from IMS
UK—Scotland	Taxation	37,340	9.1	Prescribing Information Systems (PIS) from NHS National Services Scotland Corporate Warehouse

The region of Catalonia is included as it is difficult to obtain comprehensive drug utilization data from across Spain, and Catalonia is one of the principal autonomous communities in Spain, which has been active over a number of years with initiatives to improve the quality and efficiency of prescribing (Coma et al., 2009; Björkhem-Bergman et al., 2013). Tayside was also included, representing a region in Scotland, since at the time it was difficult to obtain drug utilization data from across Scotland.

The article "Introduction and Utilization of High Priced HCV Medicines across Europe; Implications for the Future" was published in 2016. Journal: Front Pharmacol.

### Utilization data

Utilization data were collected in Defined Daily Doses (DDD)^16^, with Table 3 providing details of the DDDs used.

**Table 3:** **DDDs for medicines to treat Hepatitis C^15^**.

**Medicine**	**ATC**	**DDD**
Bocepravir (BCV)	J05AE11	2.4 g (oral)
Peg-interferon alfa-2a	L03AB11	26 mcg (parenteral)
Peg-interferon alfa-2b	L03AB10	7.5 mcg (parenteral)
Ribavirin	J05AB04	1 gm (oral)
Telaprevir (TVR)	J05AE11	2.25 gm (oral)

Population data from Eurostat were used to calculate DDDs per 1000 inhabitants per quarter (DIQs)^17^. Calculations were performed using the quarterly time period since the treatment period for HCV treatments is at least 12 weeks, and mostly 24 or 48 weeks, thereby providing a realistic denominator.

Results were calculated using two approaches. Firstly, the utilization of BCV and TVR was calculated separately to compare their uptake across countries. Due to the lack of patient specific data and different algorithms for BCV and TVR, their utilization was not combined. The second approach was an estimation of percentages of treated patients with triple therapy (ribavirin + pegIFN + TVR + BCV) vs. dual-therapy (ribavirin + pegIFN). This was again because we did not have access to individual patient data nor to prevalence rates. The percentage of treated patients was estimated through assessing the utilization of BCV and TVR in relation to ribavirin. Ribavirin is used as a proxy for dual-therapy because it is typically administered with pegIFNs, although we are aware that some patients with GT3 may be administered ribavirin without pegIFN. We acknowledge that there are differences in GT1 prevalence rates among European countries (Cornberg et al., 2011; Deuffic-Burban et al., 2012), that treatment algorithm data are not always available and there are different opinions and barriers to care (McGowan et al., 2013). Differences in GT1 prevalence rates and current treatment approaches are the most important uncertainties in this analysis. Consequently, we made a number of caveats to give a more realistic approach.

Estimates for GT1 is between 35 and 75% (Cornberg et al., 2011; Deuffic-Burban et al., 2012) of patients with chronic HCV (Table 1). In our approach, we used 45–65% to give a reasonable perspective. TVR treatment length varies between 12 of 48 weeks (25%) for patients with cirrhosis to 12 of 24 weeks (50%) for patients without cirrhosis and early SVR responses. For BCV, treatment length varies between 32 of 48 (67%) weeks for some treatment naïve patient without cirrhosis, mainly relapsers and partial responders, and 44 of 48 (92%) weeks for patients with cirrhosis (Christensen et al., 2012; Hofmann et al., 2012; Lagging et al., 2012; Leroy et al., 2012; Orlent et al., 2012; Ramachandran et al., 2012)^1, 2^. Sixty five and forty five percent GT1 prevalence rates were combined with percentages of treatment length, e.g., for TVR this was 25% use and 45% GT1 prevalence (25% of 45%) equating to 11.25%. Subsequently, the numbers used to estimate the potential for triple therapy are between 11.3 and 32.5% utilization for TVR and 30.2 and 59.7% utilization for BCV (Table 4). These findings define the second approach in an attempt to estimate the number of patients receiving triple therapy as a percentage of all HCV treated patients.

**Table 4:** **Calculated percentages for triple therapy vs. all HCV treated patients**.

**GT1 prevalence**	**Treatment length for TVR between 25 and 50% of full treatment**	**Treatment length for BCV between 67 and 92% of full treatment**
45% GT1 prevalence	11.3–22.5%	30.2–41.4%
65% GT1 prevalence	16.2–32.5%	43.5–59.7%

The article "Introduction and Utilization of High Priced HCV Medicines across Europe; Implications for the Future" was published in 2016. Journal: Front Pharmacol.

### Reimbursement expenditure data

Reimbursement expenditure was calculated in Euros per DDD (EUR/DDD). Exchange rates for Croatia, Denmark, Poland, Sweden and Switzerland where pertinent were calculated using the following conversion rates (conversion date 1-January 2008 as this was the start of the data collection period): 1 EUR = 7.6 HRK (Croatian Kuna), 7.46 DKK (Danish Krone), 9.44 SEK (Swedish krona), 1.65 CHF (Swiss franc), and 3.60 PLN (Polish zloty)^18^.

### Descriptive review of national and regional health authority demand-side activities regarding HCV drug treatment for BCV and TVR

Measures undertaken by health authorities to potentially influence the subsequent utilization of BCV and TVR were collected and collated using the 4E—Education, Engineering, Economics, and Enforcement (Wettermark et al., 2009) methodology. This method was developed in order to make it easier to understand and compare the complexity and multiplicity of healthcare policies across countries and their potential impact and/or influence (Coma et al., 2009; Wettermark et al., 2009; Godman et al., 2010a,b; Godman et al., 2013b, 2014a; Garuoliene et al., 2011; Vonèina et al., 2011; Malmström et al., 2013). Table 5 shows definitions and gives some examples of the four dimensions.

**Table 5:** **Description 4E method—Education, Engineering, Economics, and Enforcement (Garuoliene et al., 2010; Godman et al., 2010a,b, 2014b, 2015; Maticic, 2014; Moon et al., 2014; Putrik et al., 2014; Campbell et al., 2015)**.

**Approach**	**Description and examples**
Education	• Activities include educational programmes that influence prescribing: e.g., national and regional guidelines with inclusion criteria, monitoring requirements, EBM initiatives (rational prescribing), and benchmarking (quality control), e.g., monitoring of prescribing against agreed guidance coupled with feedback, e.g., “Wise list” in Stockholm, Sweden
	• Activities also include education for patients including public awareness through campaigns, world hepatitis day, flyers/printed material, as well as prescribing guidance for patients to enhance patient-doctor communication
Engineering	• This refers to organizational or managerial interventions
	• Activities include programs and interventions to optimize prescribing: e.g., structured programmes to optimize the entry of new medicines, price: volume agreements, capping budgets, and prescribing targets
	• In addition any disease management programmes to optimize treatment including potential quality targets
Economics	• Activities include positive and negative financial initiatives for all key stakeholder groups
	• Examples include percentage reimbursement/patient co-payment levels as well as financial incentives for physicians
Enforcement	• Activities include regulations such as those enforced by law; e.g., prescribing restrictions including designated signatures on prescription forms, prior authorization schemes and compulsory agreements such as compulsory international non-proprietary name (INN) prescribing and compulsory generic substitution

Country data were collected through an interactive and iterative process. Answers to the developed questionnaire were provided in written format by the co-authors, and subsequently checked for accuracy. Alternatively, country profiles were provided by one of the co-authors (Winnie De Bruijn) based on published sources as well as web-based articles. As a result, more European countries were included in the country profiles of ongoing activities regarding BCV and TVR than provided utilization data. Subsequent answers were re-checked and re-confirmed with the co-authors to enhance the robustness of the country profiles. This method has been used in previous publications involving health authority personnel (Garuoliene et al., 2010, 2011; Godman et al., 2010a,b, 2013b, 2014a,b; Vonèina et al., 2011; Malmström et al., 2013); consequently, applied in this research project.

The article "Introduction and Utilization of High Priced HCV Medicines across Europe; Implications for the Future" was published in 2016. Journal: Front Pharmacol.

All country profiles were supplemented with data from the WHO Hepatitis report^19^ and Euro Hepatitis Index 2012 report (Cebolla and Björnberg, 2012).

Patient consent as well as ethics approval was not required as aggregate utilization and expenditure data were obtained from anonymised health authority databases (Table 2). This is in line with previous publications involving anonymised aggregated health authority data Europe (Godman et al., 2010a, 2014a; Vonèina et al., 2011; Moon et al., 2014).

## Results

### General

In the majority of countries studied, both BCV and TVR were reimbursed. Exceptions included Bosnia and Herzegovina as well as Estonia (Table 6). Technically in Sweden only TVR is included in the national reimbursement scheme. However, in practice, both BCV and TVR are free for patients as both medicines are free for infectious diseases under the Infectious Disease Act.

**Table 6:** **Summary of most important demand side measures among European countries to influence the prescribing of BCV and TVR post-launch**.

**Country**	**4E**	**Approach**
Austria	Enforcement	• Prior authorization scheme with cost-sharing for TVR
	Engineering	• PIs are reimbursed according to the published “limitations of prescription”—as long as a patient meets the criteria defined in the “limitations of prescription” his/her treatment will be approved and thus reimbursed
		• No reimbursement of BCV for null responders
Belgium	Enforcement	• Need prior approval from the Health Insurance companies according to agreed criteria (chapter IV medicine) before PIs can be used.
		• Otherwise, 100% patient co-payment if prescribing does not follow agreed criteria
Bosnia and Herzegovina (Republic of Srpska)	Education	• Guidelines available for the diagnosis and treatment of chronic hepatitis C
		• Increasing public awareness as well as campaigns stating that there is free, voluntarily, anonymous testing and counseling for patients with suspected HCV. Alongside this, distribution of educational materials—helped by establishing counseling centers for hepatitis and HIV
	Economics	• Therapy initiated only in specialist centers for patients with hepatitis
	Engineering	• Health Insurance Fund purchases medicines for patients with HCV under a 1-year (centralized tender) with defined reimbursement conditions; otherwise 100% co-payment
	Enforcement	• However, neither BCV (market authorization in B&H in 2012) or TVR (no application so far submitted in B&H) are currently reimbursed (100% co-payment); so far (March 2016) there have been no requests for a refund sent to the Health Insurance Fund
		• Proposed wholesale price by the manufacturer within the market authorization process was €4720/package
Croatia	Engineering Enforcement	• Incidence and prevalence of HCV has been declining in Croatia in recent years through preventative measures. These include ensuring safety of blood products, reducing drug abuse as well as programs to reduce infection rates among intravenous drug users
		• Both BCV and TVR are reimbursed and on the list of expensive products since 2013 (BCV in Official Gazette 49/2013 and for TVR in Official Gazette 67/2013)
		• They are both reimbursed for triple therapy but with defined guidance for use for reimbursement. Treatment is reimbursed only in hospitals to ensure prescribing is in line with current guidelines/guidance
France	Education Engineering Enforcement	• The prevention and management of HCV has been on the public health agenda in France since the early 1990s, with an extensive network of hepatologists and reference centers
		• The authorities through the referral centers also research outcomes from current treatment approaches
		• Only physicians specialized in hepatology, internal medicine or infectious diseases are allowed to initiate treatment with DAAs including BCV and TVR
Iceland	Education	• Both BCV and TVR are reimbursed
		• Guidelines are available but currently no health authority activities directing prescribing
		• More recently a nationwide treatment-project where all HCV infected patients are being offered the second generation DDA's over a 2–3 years period.
		• Alongside this, a large scale epidemiological study is ongoing to ascertain whether it is possible eliminate HCV from a small, relatively confined population such as Iceland
Ireland	Education Engineering Economics Enforcement	• Surveillance system in place to collect effectiveness, safety, tolerability and economic outcomes from current treatments including BCV and TVR
		• All patients prescribed triple therapy are obliged to be registered with the Irish Hepatitis C Outcome and Research Network (ICORN) treatment database which captures longitudinal data
		• Dispensing of BCV and TPR is restricted to hospitals only to ensure appropriate governance of treatment
Italy	Education Engineering Economics Enforcement	• Italian Horizon Scanning group issuing information on medicines for patients with chronic HCV to national and regional authorities
		• Price volume agreements - if expenditure on BCV and TVR exceeds pre-set thresholds, manufacturers payback any differences to the Italian National Health Service
		• As a result, BCV has a patient cap of 6000 patients for 2 years and a sales cap of €120 million/year and 5% discount with pegIFN. TVR has a patient cap of 2000 patients the first year, 3000 patients for the second year and re-negotiation above 4000 patients. Sales cap of €100 million/per year. Re-negotiation above €80 million per year^21^
		• Physicians need to be validated by the Italian Medicines Agency with only selected centers and physicians allowed to prescribe treatment.
		• In the Veneto Region, a special network of centers exists to administer HCV medicines
		• Patient registers are in place for patients receiving PI to monitor their use according to agreed guidance (and increasingly monitor outcomes in the future). Patient entry encouraged as part of the payment system for hospitals; otherwise hospitals will not reimbursed for the medicines costs for patients with HCV
Malta	Economics, Enforcement	• Treatments initially were not reimbursed by the National Health Service. Some patients bought their treatment privately or were supported through NGOs. Alpha interferon was originally used and later pegylated interferon and ribavirin became standard treatments in Malta (Brincat et al., 2013)
		• Subsequently, a one-time donation of medicines was undertaken by pharmaceutical companies enabling some patients to be initiated with ledipasvir/sofosbuvir
		• Recently, newer treatments including sofosbuvir were included in the National Formulary List to be provided free of charge through the National Health Service. Their use is regulated by protocols approved by the HCV Patient Management Committee
Netherlands	Enforcement	• Need prior approval according to agreed guidance before a PI can be dispended
Slovakia	Enforcement	• To be eligible for reimbursement, a psychiatrist must make a statement that drug abusers are abstinent for at least 1 year
Slovenia	Education Engineering Enforcement	• Detailed patient register schemes which include additional data for prescribing a PI: fibrosis stage, IL28B type, prior HCV treatment, type of PI included in treatment, lead-in phase and rapid virological response
		• When patients with HCV are treated, data is added according to the national protocol for the management of HCV in patients with HCV. The registry was established in 2007
		• Slovenia has a National Viral Hepatitis Expert Group since 1997, established to develop national treatment guidelines and evaluate the efficacy and safety of different treatment approaches in clinical practice
		• Since 1997, there is a national network of a named list of infectologists and hepatologists in 5 reference centers for treatment of viral hepatitis. These are the only physicians who can prescribe HCV therapy (in accordance with the national guidelines)
		• Since 2007, there is an interdisciplinary National healthcare network across the country for the treatment of HCV in patients who inject themselves with drugs
		• The Health Insurance Institute of Slovenia (ZZZS) has a possibility to control physician prescribing where regulations exist. When prescribing is not in line with prescribing restrictions, the provider physician/hospital has to pay a fine
Spain—Catalonia	Education Engineering Economics	• Available algorithms of chronic HCV treatment at a national and regional level, including IL28B testing as well as selection of dual or triple therapy in naïve/relapsers/non-responder patients
		• Register of prevalence and treatment outcomes ongoing
		• Data from surveillance systems are used to regularly monitor expenditure and benchmarking among hospitals. Also monitoring of erythropoiesis factor requirements (management and impact of side effects)
		• PI related data incorporated into the surveillance system. This includes the numbers of patients treated for HCV treated with a PI, which PI and PegIFN is selected as well as co-infected patients with HIV and organ transplanted patients treated with a PI
		• It is recommended a multidisciplinary treatment approach is undertaken to improve care including for instance a gastroenterologist/infectious disease physician, psychiatrist, pharmacist and laboratory testing personnel
		• Annual budgets for outpatient drug treatments are allocated to Catalan public hospitals (including drugs for cancer, HCV, multiple sclerosis, etc.) to help control costs
		• There are currently no patient co-payments for HCV medicines in Catalan public hospitals
Sweden	Education Engineering Economics	• National treatment guidelines available to guide treatment
		• BCV is currently not reimbursed by the TLV (Dental and Pharmaceutical Benefits Agency - reimbursement authority in Sweden) but TVR is. However, all drugs for HCV infection, including TVR and BCV, are free for the patient since medicines for infectious diseases including Hepatitis C are free under the Infectious Diseases Act
		• TVR is currently reimbursed without restriction
Turkey (Aygen et al., 2015)	Engineering Enforcement	• BCV and TVR are reimbursed with restricted indications, e.g., triple therapy is reimbursed in combination with TVR in patients infected with HCV genotype 1 who have compensated liver disease and who have previously received PegIFN/RBV therapy and relapsed
		• In patients with compensated liver disease, total treatment duration is 48 weeks with 12 weeks of TVR therapy, provided that the liver biopsy Ishak score is stage ≥4, the platelet count is below 100,000/mm^3^, or the prothrombin time is over 3 seconds
		• In relapsed patients, total treatment duration is 24 weeks, including 12 weeks of TVR therapy if HCV RNA is negative at week 4 of treatment, and 48 weeks if HCV RNA is positive at week 4 of treatment
UK—Scotland	Engineering	• Pro-active approach to the introduction of triple therapy including BCV and TCR
		• Patient numbers are tracked to check they agree with original predictions and the case for funding (in Tayside)

NB. BCV, Boceprevir; DAAs, direct acting antivirals; pegIFN, pegylated interferon; PI, Protease inhibitor; TVR, Telaprevir. Estonia is not included in the Table as the pharmaceutical companies were providing first generations DAAs free of charge until recently.

The article "Introduction and Utilization of High Priced HCV Medicines across Europe; Implications for the Future" was published in 2016. Journal: Front Pharmacol.

### Activities among by health authorities to influence the prescribing of BCV and TVR

Table 6 summarizes the variety of measures broken down by the 4E method (Table 5) implemented by the various European countries to improve the management of patients with HCV. This includes any measures regarding subsequent utilization of BCV and TVR.

All European countries studied had a national strategy plan to manage patients with HCV, which typically included prevention and control programmes and/or guidelines^19^. All clinical guidelines available in English typically followed the strict EMA recommendations, e.g., besides SVR monitoring, there were also clear starting and stopping rules prior to initiating treatment and continuing treatment (European Association for the Study of the Liver, 2011; Hofmann et al., 2012; Lagging et al., 2012; Leroy et al., 2012; Orlent et al., 2012; Ramachandran et al., 2012)^1, 2^. Where countries mostly differed was their opinion regarding genotyping interleukin 28B (IL28B) polymorphism. Some countries and regions recommend routine testing, e.g., Catalonia, whilst others currently do not test.

All countries studied had a surveillance system for either acute and/or chronic HCV infections. Unfortunately current registries are heterogeneous and differ mostly in case definition (European Centre for Desease Prevention Control, 2010; Cornberg et al., 2011; Yehia et al., 2014)^20^. The EMA Committee for Medicinal Products for Human Use (CHMP) emphasized that the prescribing of BCV and TVR must be undertaken by professionals with knowledge and experience of HCV, including testing and treatment^1, 2^. Consequently, triple therapy must be prescribed by doctors who specialize in HCV management^1, 2^. This is typically the case for BCV and TVR, which are only licensed for GT1. This means physicians are obliged to test for genotypes before starting treatment.

All European countries that reimbursed triple therapy typically had no patient co-payment. We are aware that risk sharing agreements and discounts are used by health authorities to control budgets, enabling patients to have access to new high priced medicines (Adamski et al., 2010; Ferrario and Kanavos, 2013). However, data on the extent of any discounts are typically lacking as such arrangements are confidential. As a result, we were unable to document any cost/DDD data for BCV and TVR in Scotland (Tayside). Reimbursement for HIV co-infection and treatment before and after liver transplantation currently exists in a number of European countries including Austria, Ireland, Catalonia, Scotland, Slovakia, Slovenia and Sweden.

### Utilization

The uptake of BCV and TVR varied between the countries and over time (Figures 1A,B). The highest uptake for TVR was in Tayside (Scotland) in the second quarter of 2012 at 2.4 DIQs. The highest uptake of BCV was in Belgium at 1.32 DIQs. Subsequently all countries showed a decrease of HCV medicines between approximately 6 months after triple therapy reimbursement, e.g., the Netherlands, Belgium, and Slovenia, and 12 months after triple therapy reimbursement, e.g., Austria, Denmark, Catalonia and Sweden. Utilization of BCV was highest in Belgium with 38% in third quarter after reimbursement (Q1 2013) and lowest in Italy and Estonia.

**Figure 1:** **Uptake BCV and TVR across European countries from the month first reimbursed**. Each Bar represents a 3 month period. Only the first quarter of 2012 and 2013 is displayed in the legend to include all countries. **(A)** Included countries are: AU, Austria; BE, Belgium; DK, Denmark; EE, Estonia; ES (CT), Catalonia (Spain). **(B)** Included countries are: IT, Italy; NL, the Netherlands; UK-Scot (TS), Tayside (Scotland); SI, Slovenia; SE, Sweden; TR, Turkey.

The article "Introduction and Utilization of High Priced HCV Medicines across Europe; Implications for the Future" was published in 2016. Journal: Front Pharmacol.

The upper and lower range (dotted lines in Figures 2, 3) illustrate the utilization of BCV and TVR if all potential patients with GT1 prevalence of 45–65% were treated (see comments in Table 4). For TVR, only Sweden meets the upper limit, which equates to the 65% GT1 prevalence and greatest percentage of therapy containing TVR. Only Austria, Estonia, Italy, and Catalonia do not meet the lower limit, indicating that even in a hypothetical situation with low GT1 prevalence and a short DAA treatment length, not all patients who should receive triple therapy actually receive it. For BCV, Belgium touches the lower limit with lowest GT1 prevalence and a lowest percentage of treatment containing BCV. Due to lack of patient specific data, prevalence data and different algorithms, the utilization of BCV and TVR are not consolidated. However, after adding BCV and TVR together, Belgium, Denmark, the Netherlands and Sweden appear to have the highest uptake of triple therapy vs. dual therapy.

**Figure 2:** **Percentage utilization of TVR vs. ribavirin in quarters following reimbursement**. NB: Upper range genotype 1 prevalence (=GT1) is 65% and highest percentages (50%) triple therapy containing TVR (mostly non-cirrhotic patients). Lower range GT1 prevalence is only 45% and lowest percentages (25%) triple therapy containing TVR (mostly cirrhotic patients).

**Figure 3:** **Percentage utilization of BCV vs. ribavirin in quarters following reimbursement**. Upper range genotype 1 prevalence (=GT1) is 65% and highest percentages (92%) triple therapy containing BVC (mostly cirrhotic patients). Lower range GT1 prevalence is only 45% and lowest percentages (67%) triple therapy containing BVC (mostly naïve non-cirrhotic patients).

### Expenditure data

Table 7 contains reimbursed expenditure/DDD data for both BCV and TVR up to May 2013. Turkey was excluded as only IMS data were available. Estonia was excluded as these medicines have only recently been reimbursed, and Scotland (Tayside) was excluded as reimbursed data included confidential discounts; consequently unavailable for analysis. There were no differences in the documented prices between medicines dispensed in hospital pharmacies for out-patients or community pharmacies. However, this did not include any confidential discounts as part of risk sharing or other agreements (Adamski et al., 2010; Ferrario and Kanavos, 2013; Vogler et al., 2013).

The article "Introduction and Utilization of High Priced HCV Medicines across Europe; Implications for the Future" was published in 2016. Journal: Front Pharmacol.

**Table 7:** **Reimbursed Euro per DDD (EUR/DDD) from the time of reimbursement until the latest available data (May 2013) of TVR and BCV**.

	**Telaprevir (TVR)**		**Boceprevir (BCV)**	
	**EUR/DDD when reimbursed**	**EUR/DDD 05-2013**	**EUR/DDD when reimbursed**	**EUR/DDD 05-2013**
Austria^*^	321.48	310.44	146.60	116.11
Belgium^*^	324.58	324.54	116.66	116.66
Belgium^**^	315.29	–	113.31	–
Croatia^**^/^***^	331.97	331.97	123.46	123.46
Denmark^**^	394.65	384.53	145.53	131.62
Netherlands^*^	300.23	302.66	114.51	114.05
Slovenia^*^	302.31	291.64	113.10	113.10
Spain-Catalonia^**^	304.74	304.74	103.92	103.92
Sweden^*^	329.49	294.82	117.69	118.52

NB:

* Dispensed in community pharmacy;

** Dispensed in hospital pharmacy;

*** Price from basic list and price from expensive product list (same prices). Reimbursed prices of BCV and TVR should not be compared as different treatment paradigms.

For both BCV and TVR, Denmark appeared to pay the highest reimbursed price at 131.52 and 384.53 EUR/DDD respectively. Catalonia (Spain) appeared to pay the lowest reimbursed price at 103.92 EUR/DDD for BCV and Slovenia the lowest reimbursed price for TVR at 291.64 EUR/DDD. Only Austria had a major price decrease from EUR 146.60 to EUR 116.1 per DDD during the course of the study following agreements.

Total expenditure for HCV treatments was decreasing in all countries before the reimbursement of BCV and TVR, especially in Catalonia and Austria (Figure 4), and again prior to the availability of the newer second generation DAAs, at the end of 2012 and beginning of 2013. Denmark and Slovenia had the lowest increase in EUR/1000 inhabitants/3 months after the reimbursement of BCV and TVR. This was 99 and 89% respectively between the lowest and highest EUR/1000 inhabitants/3 months from just before impending reimbursement of these two medicines to just after. This compares with a rise of 385% in Catalonia.

**Figure 4:** **Expenditure on treatments for HCV (Euro/1000 inhabitants/quarter) from 2008 to 2013**. NB: ◯ = reimbursement agreed BVC. Sweden and Denmark first quarter after EMA approval are included.

## Discussion

Our analysis showed reasonable consistency in the uptake of BCV and TVR among the European countries studied (Figure 1) compared with appreciable differences that have been seen in the utilization of new high priced medicines to treat patients with rheumatoid arthritis, type 2 diabetes and cancer across Europe (Hoebert et al., 2012; Jönsson et al., 2014; Putrik et al., 2014; Nolte and Corbett). This is despite appreciable differences among the participating countries in their level of spending on healthcare as well as the percentage of GDP they spend on health (Table 1). This might be explained firstly by the fact that all European countries followed EMA labeled indications with strict regulations for clear genotyping and SVR monitoring. Secondly, there were relatively few measures implemented among European health authorities to influence physician prescribing of either BCV or TVR apart from directing prescribing to specialists and specialist centers and entering patients into registries. Thirdly, both treatments were typically 100% reimbursed although there are exceptions (Table 6).

The article "Introduction and Utilization of High Priced HCV Medicines across Europe; Implications for the Future" was published in 2016. Journal: Front Pharmacol.

The rapid uptake of BCV and TVR across countries (Figure 1) may be explained by expectancy among professionals and patients regarding the increased efficacy of these first generation DAAs vs. previous regimens. This resulted in countries placing patients on waiting lists to receive triple therapy soon after BCV and TVR were reimbursed. Whilst we cannot say this with certainty, this is in line with decreasing costs of ribavirin and pegIFNs before reimbursement of the new PIs (Figure 4). Additionally, European guidelines advised postponing HCV treatment until the new DAAs including sofosbuvir became available in view of their greater efficacy and tolerability as well as reduced length of treatment (European Association for the Study of the Liver, 2011; Hatzakis et al., 2011).

The consistency in the utilization of BCV and TVR across Europe appears promising, especially considering a desire to reduce infection rates whilst attempting to keep the budgets for these medicines manageable. Any differences in utilization rates of BCV and TVR between countries (Figure 1) could potentially be explained by differences in HCV and GT1 prevalence variations as well as local physician preferences and knowledge rather than any specific health authority interventions (Table 6). However, we cannot comment further as we did not have access to patient level data. In addition, we did not explore key issues among specialist physicians involved in the management of patients with HCV.

Reimbursed prices for BCV and TVR (EUR/DDD) also appeared comparable among the European countries studied. This did not include risk-sharing agreements including rebates and discounts as information about these agreements is limited, with the exception of Italy. This is because such measures are typically confidential.

The upper and lower ranges identified in Figures 2, 3 suggest that the uptake of triple therapy appears reasonable in a number of the studied countries based on the assumptions of GT1 prevalence and treatment algorithms (Table 4); although, lower in some countries. However, there needs to be caution when interpreting these results as a number of assumptions were made (Table 4), and we are aware of the concerns with current estimated prevalence rates for HCV GT1 (Table 1). Utilization data can also be complicated by other factors, which include patients being selected for dual therapy if they have a low HCV RNA viral load after 4 weeks or ILB28B favorable CC polymorphism. Analysis of subsequently available patient level data in Stockholm, Sweden, showed that among patients initiated on treatment in 2012, total (TVR+BCV)/ribavirin was approximately 64% in 2012, which corresponds to Figures 2, 3 (Frisk, Personal Communication). However, in Catalonia, TVR+BCV/ribavirin was used in approximately 18.6% of patients, which is higher than in our study (Ibáñez, Personal Communication). In a recent report involving Italy, France, Germany, Spain and UK, most gastroenterologists stated that triple therapy would be prescribed more for non-responders in the first year of its availability. By 2014, 60% of treatment-naïve patients were expected to be treated with triple therapy^22^. This wide predicted variation in the prescribing of DAAs was not seen in practice (Figures 1A,B), with the utilization of BCV and TVR (Figures 1A,B) appearing more similar compared with the appreciable differences in the utilization of other high priced medicines, e.g., TNF alpha inhibitors and those to treat patients with cancer or Type 2 diabetes (Hoebert et al., 2012; Jönsson et al., 2014; Putrik et al., 2014; Nolte and Corbett).

The article "Introduction and Utilization of High Priced HCV Medicines across Europe; Implications for the Future" was published in 2016. Journal: Front Pharmacol.

One reason for the lower than expected surge in the use of triple therapy in Europe could be that efficacy and safety data from clinical trials are not always replicated in clinical practice and side effects can be more frequent and severe. This is especially the case in treatment-experienced HCV patients as observed in the French cohort reported by Hézode et al. (2013, 2014). The same phenomenon has been seen in Ireland where the effectiveness in patients entered into the registry (Table 6) was considerably lower than those seen from the clinical trials (O'Leary, Personal Communication). Published studies in the US have shown that the uptake of triple therapy was also relatively low, although TVR (INCIVEK®) reached 1 US$ billion within a short time and US$1.6 billion after the first year^23^. In a small study (487 GT1 patients), only 18.7% of patients received triple therapy in the first year after FDA approval (Chen et al., 2013). Reasons not to start triple therapy were principally contraindications (50%). Of all the patients who started triple therapy, 21% discontinued it. This was mostly because of side effects (Chen et al., 2013). Other studies have also concluded that side effects are the most frequent barrier for chronic HCV treatment (McGowan et al., 2013)^.^

The article "Introduction and Utilization of High Priced HCV Medicines across Europe; Implications for the Future" was published in 2016. Journal: Front Pharmacol.

Consequently, side effects and complexity of drug treatment posology of PIs may explain the decrease in utilization and expenditure of BCV and TVR in recent years among European countries (Figures 1, 4) coupled with the anticipation of the new second generation DAAs, with less side effects, shorter treatment durations, the potential for interferon free regimens and the potential for cures (Brennan and Shrank, 2014; Kohli et al., 2014)^3^. We are aware for instance that in Catalonia, France and Sweden, a number of potentially eligible patients for BCV and TVR were put on waiting lists until the launch of the second generation DAAs, and probably in other countries as well.

This observation is strengthened by recent findings showing that sofosbuvir, after TVR, was the fastest growing prescribed medicine in the US with sales of US$2.27 billion in the first quarter of 2014^24^ reaching, as mentioned, US$12.4 billion worldwide in 2014. This accounted for 37.5% of expenditure on HCV medicines among managed care organizations in 2014 (Trooskin et al., 2015)^11^. This expenditure is helped by the cost of a standard 12-week course of sofosbuvir and simeprevir being initially at US$84 000 and US$66,000 in the US respectively, with sofosbuvir initially priced at between Euro 50,000 and 60,000 per 12-week course among Eurozone countries, although U$54,000 (€44,000) in the UK and €41,000 in France (Brennan and Shrank, 2014; Lemoine and Asia, 2014; Phelan and Cook, 2014; van de Ven et al., 2014; Trooskin et al., 2015; Iyengar et al., 2016). These prices, coupled with the prevalence of HCV, have already resulted in activities among countries to control costs through price negotiations and other strategies. This is not surprising with potential sales of US$15 trillion if an estimated 180 million people worldwide with HCV were treated with sofosbuvir (Montazerhodjat et al., 2016). Table 8 summarizes some of the activities, exacerbated for instance by the authorities in France initially being charged sofosbuvir at 756 times the cost of its production in France (Phelan and Cook, 2014).

**Table 8:** **Price negotiations and other strategies across countries to reduce the expenditure burden of second generation DAAs**.

**Country**	**Summary of ongoing pricing negotiations across countries**
Australia	• Ongoing schemes in Australia to enable access to new effective DAAs, including potential pricing policies, as the proposed budget impact of over Australian $3 billion over a 5 year period is considered unaffordable^25^
Brazil	• Negotiated prices for sofosbuvir are as low as US$7000/12-weeks treatment course^26^
	• Negotiated price for a bottle (28 capsules) of simeprevir in Brazil is US$1000 (Andrieux-Meyer et al., 2015)
	• BCV and TVR now removed from the public funded (SUS) treatment programmes in view of their lower effectiveness and greater side-effects compared with the second generation DAAs
Egypt and India (Brennan and Shrank, 2014; Phelan and Cook, 2014; Trooskin et al., 2015)	• Egyptian authorities negotiated a 99% discount of the US price—bringing its price in Egypt down to US $900 per 12-week course
	• Sofosbuvir is being manufactured in India at a cost of < US$250/course as Gilead was denied a patent in India
France	• Second generation DAAs were initially only reimbursed for advanced liver fibrosis (F2-F4) (Dedet, Personal Communication)
	• More recently, the government in France introduced a new tax using a “progressive contribution scheme”
	• As a result, the Economic Committee for Health Products agreed a price of €13,667 per 28-tablet pack for sosfobuvir alone, i.e., approximately €5000 lower than the initial list price, at an overall negotiated price of €41,000 (US$51,000) for a 12-week course
	• Prices are likely to fall further with the launch of additional DAAs to help cure patients with HCV^27^, including the combination of sofosobuvir and ledipasvir leading to a potential cure initially at €48,000/treatment course^28^. The negotiated price for sofosbuvir+ ledipasvir was finally set at €547.619 per tablet, i.e., €46,000/treatment course^29^
Georgia^30^	• The minister of health, labor and social affairs in Georgia emailed Gilead to say they had a fund of US$5 million to help eradicate HCV with an infection rate of almost 7%
	• Gilead subsequently agreed to provide sofosbuvir free of charge to help eliminate the disease within 10 years
Italy	• The Italian Reimbursement Agency (AIFA) negotiated a price reduction scheme with the reimbursed price for “initial patients” at €37,000/patient/course dropping to €4000 for the “last” patients, averaging €18,000 per patient (Messori, 2015a)^31^
	• As a result, overall expenditure for sofosbuvir in Italy is expected to be less than €500 million per year initially, which was acceptable to all^30^
South Africa^32^	• Access to hepatitis treatment in South Africa remains limited due to a combination of patent, registration and cost barriers
	• More recently, Gilead is allowing the importation of the fixed-dose combination treatment, HARVONI, with a preferential pricing for the public sector at just one one-hundredth of the US price, i.e., approximately R17,000 for a 12-week course
Spain	• The negotiated price per course is approximately US$25,000 per course (EU 20,500) or lower, with the ministries of Health and Finance agreeing with the regional health ministries to establish a funding plan to ensure all eligible patients will be treated with the second generation DAAs for at least 12 weeks
	• In addition, the health outcomes of patients will be assessed (Trooskin et al., 2015)^33^. Overall, a national expenditure ceiling of Euro727 million euros has been established to fund these new treatments for patients with HCV in Spain^32^
Sweden	• Risk sharing arrangements to lower prices has resulted in improved access among the County Councils (Regions—budget holders)
	• Alongside this, the authorities in Sweden are currently monitoring the effectiveness (viral load) and safety of second generation DAAs in routine clinical care
USA	• Private Insurance Plans (Managed Care Organizations—MCOs) have included sofosbuvir in their formularies although a number of MCOs have included coverage alongside prior authorization (PA) to conserve resources
	• Encouraging the use of second generation DAAs irrespective of the METAVIR score, along with PA schemes to encourage 8 weeks of treatment, has resulted in a plateau or fall in usage, endorsing this approach
	• MCOs alongside pharmacy benefit management (PBM) schemes have also established data registries to track patient outcomes in terms of relapses and/or reinfection rates
	• Among most State Medicaid schemes, patients must have a METAVIR score of F3 or F4, indicative of severe liver disease, to receive sofosbuvir
	• 30 States also require sofosbuvir to be prescribed by, or in consultation with, a specialist such as a hepatologist, gastroenterologist, or infectious disease physician before funding, and some States have introduced a sobriety requirement (Canary et al., 2015; Rein, 2015; Trooskin et al., 2015).
	• Proposals for new methods to finance such transformative therapies through healthcare loans and securitization (Montazerhodjat et al., 2016)

There are also ongoing activities among other African countries including Botswana and Zimbabwe given the higher prevalence of HCV in developing countries and the potential for generic agreements. These differences in policies for the second generation DAAs is already leading to considerable differences in their utilization rates in Europe^34^.

The article "Introduction and Utilization of High Priced HCV Medicines across Europe; Implications for the Future" was published in 2016. Journal: Front Pharmacol.

Recent analysis has shown there is still appreciable variation in the price of second generation DAAs across countries (Andrieux-Meyer et al., 2015). For instance, the price per bottle of sofosbuvir (28 tablets) ranges from $300 (India and Pakistan) and $402 (Nigeria—current market survey) to $20,590 in Switzerland, and for daclatasvir from $175 in Egypt and $252 in Nigeria (current market survey) to $14,899 in Germany (Andrieux-Meyer et al., 2015). Overall, prices are generally substantially lower in LMIC countries although there are outliers, with little correlation between prices and per capita income levels among higher income countries, e.g., the price for a bottle of simeprevir ranges from U$9166 in Spain to US$14,865 in Australia (Andrieux-Meyer et al., 2015).

It is likely that prices of second generation DAAs will continue falling across countries with estimates of manufacturing for 12-week courses at US$10-$30 for daclatasvir, US$68–$136 for sofosbuvir, US$100–$210 for faldaprevir and US$130–$270 for simeprevir (Hill et al., 2014) coupled with increased competition. This should also help the management of patients with genotypes 4, 5, and 6 that are mainly present in Africa, the Middle East and Asia, where resources are more limited (Papastergiou and Karatapanis, 2015). Their availability as oral therapies coupled with the potential of avoiding genotyping with its associated facilities and costs should further help with increased usage and price negotiations (Ford et al., 2014; Younossi et al., 2015).

Prices should also fall further following the inclusion of sofosbuvir, simeprevir dasabuvir and daclatasvir in the 19th edition of the WHO Model List of Essential Medicines along with comments to negotiate affordable prices^35^. This alongside the formation of consortia, which is already happening in the US with State Medicaid schemes, following the example of ARVs where prices reduced substantially following strong pressure from multiple stakeholders (Lemoine and Asia, 2014). In addition, the potential development of a Global Fund for treatments for patients with HCV or other mechanisms (Phelan and Cook, 2014).

The undoubted effectiveness of the second generation DAAs is making European and other health authorities re-think their approaches to valuing new high priced medicines. This includes new medicines for patients with cancer, as well as those for orphan diseases, which are being reimbursed at high prices despite often very limited health gain in view of patient pressure and other factors (Fojo and Grady, 2009; Hughes-Wilson et al., 2012; Experts in Chronic Myeloid Leukemia, 2013; Kantarjian et al., 2013; Simoens et al., 2013; Cohen and Felix, 2014; Ghinea et al.). This will continue and be the subject of future research projects among the co-authors. Future research will also include assessing the utilization and expenditure on second generation DAAs in clinical practice among European countries as they become standards of care (Childs-Kean and Hand, 2015), building on early analysis by the French authorities and others^33^.

## Conclusion

There appears to be reasonable consistency in the uptake and utilization of BCV and TVR among the studied European countries in comparison with other new high priced medicines. This may reflect the high social impact of chronic HCV treatment, especially with few health authority measures implemented to influence physician prescribing. However, using ribavirin as a benchmark hints at differences in the utilization of BCV and TVR. This may indicate that the prescribing of dual vs. triple therapy differs across countries. This cannot be explained by looking at health authority activities for these two treatments and may just reflect physician preference. Consequently, more information including GT1 prevalence data and data on treatment algorithms (including treatment length and treatment period containing PI) is needed to explain this.

The article "Introduction and Utilization of High Priced HCV Medicines across Europe; Implications for the Future" was published in 2016. Journal: Front Pharmacol.

There are also ongoing activities with the second generation DAAs across countries to reduce their costs in view of their undoubted effectiveness and tolerability alongside their considerable budget impact. This will be the subject of future research to provide additional guidance to authorities in the face of continuing resource pressures.

## Author contributions

WdB, CI, PF, HBP, and BG contributed to the design of the paper and the methodology. They also produced the first and subsequent drafts. AA, PVB, AB, LB, GD, JE, JOF, JF, GG, IG, AG, HG, SJ, JJ, RJ, SK, OL, NM, EM, MM, VM-P, AM, OO, AO'L, JP, CS, SS, CT, IT, MT, KT, MW, SV, EV, and CZ provided data on the utilization of BCV and TVR and/or ongoing measures within their own countries to improve the prevention and/or management of HCV. They also critiqued successive drafts of the paper. All authors read and approved the final manuscript.

### Conflict of interest statement

The authors declare that the research was conducted in the absence of any commercial or financial relationships that could be construed as a potential conflict of interest.

## Footnotes

^1^European Medicine Agency. Incivo - telaprevir [Internet]. [cited 18 Nov 2015] Available from: http://www.ema.europa.eu/ema/index.jsp?curl=pages/medicines/human/medicines/002313/human_med_001487.jsp&mid=WC0b01ac058001d124

^2^European Medicine Agency. Victrelis - boceprevir [Internet]. [cited 18 Nov 2015] Available from: http://www.ema.europa.eu/ema/index.jsp?curl=pages/medicines/human/medicines/002332/human_med_001464.jsp&mid=WC0b01ac058001d124

^3^California Technology Assessment Forum. The Comparative Clinical Effectiveness and the Value of Simeprevir and Sofosbuvir in the Treatment of Chronic Hepatitis C Infection: Final Report. San Francisco: California Technology Assessment Forum; April 15, 2014. Available at URL: http://icer-review.org/wp-content/uploads/2016/02/CTAF_Hep_C_Apr14_final.pdf (Accessed 8 July 2017).

^4^European Medicine Agency. EPAR Sovaldi sofosbuvir. [cited 2015 Nov] Available at URL: http://www.ema.europa.eu/docs/en_GB/document_library/EPAR_-_Summary_for_the_public/human/002798/WC500160599.pdf

^5^European Medicine Agency. EPAR Olysio simeprevir. [cited 2015 Nov] Available at URL: http://www.ema.europa.eu/docs/en_GB/document_library/EPAR_-_Summary_for_the_public/human/002777/WC500167869.pdf

^6^European Medicine Agency. EPAR daclatasvir. [Cited 2015 Nov]. 2014. Available from: http://www.ema.europa.eu/docs/en_GB/document_library/EPAR_-_Public_assessment_report/human/003768/WC500172849.pdf

^7^European Medicine Agency. EPAR Ledipasvir. Harvoni [Cited 2015 Nov]. Available from: http://www.ema.europa.eu/docs/en_GB/document_library/EPAR_-_Summary_for_the_public/human/003850/WC500177997.pdf

^8^European Medicine Agency. EPAR ombitasvir/paritaprevir/ritonavir. [cited 2015 Oct] Available from: http://www.ema.europa.eu/docs/en_GB/document_library/EPAR_-_Summary_for_the_public/human/003839/WC500184000.pdf

^9^Médecins Sans Frontières. THE DIAGNOSIS AND TREATMENT OF HEPATITIS C?: A technical landscape. 2013. Available at URL: http://www.msfaccess.org/sites/default/files/MSF_assets/HepC/Docs/HepC_brief_TechnicalLandscape_ENG_2013.pdf (Accessed 15 Oct 2015).

^10^Research and Markets. Hepatitis C Therapeutics Market to 2018 - Expected Launch of GS-7977 in 2015 will Pave the Way for an Oral Interferon-free Combination Therapy [Internet]. 2012. [cited 2015 Sept] Available from: http://www.researchandmarkets.com/research/ngbvll/hepatitis_c

^11^Express Scripts. The 2014 Drug Trend Report. [cited 2015 Sept]. Available at URL: http://lab.express-scripts.com/~/media/PDFs/Drug%20Trend%20Report/ExpressScripts_DrugTrendReport.ashx (Last Accessed 8 July 2016).

^12^EFPIA. HEALTH and GROWTH - Evidence Compendium. October 30th, 2013. Available from URL: http://www.efpia.eu/uploads/Modules/Documents/health-and-growth_evidence-compendium.pdf

^13^WHO. Access to new medicines in Europe: technical review of policy initiatives and opportunities for collaboration and research. Available at URL: http://www.euro.who.int/en/health-topics/Health-systems/medicines/publications2/2015/access-to-new-medicines-in-europe-technical-review-of-policy-initiatives-and-opportunities-for-collaboration-and-research.

^14^Health expenditure, total (% of GDP) - World Health Organization Global Health Expenditure database [Internet]. [cited 2015 Aug 17]. Available from: http://data.worldbank.org/indicator/SH.XPD.TOTL.ZS

^15^ATC/DDD Index 2013 [cited 2015 Sept]. Available from: http://www.whocc.no/

^16^World Health Organization (WHO). Introduction to Drug Utilization Research World Health Organization WHO International Working Group for Drug Statistics Methodology, Collaborating Centre for Drug Utilization Research and Clinic. 2003. [cited 2015 Oct]. Available at URL: http://www.who.int/medicines/areas/quality_safety/safety_efficacy/Drug%20utilization%20research.pdf

^17^Eurostat. Population on 1 January. [cited 2015 Sept] Available from: http://epp.eurostat.ec.europa.eu/tgm/table.do?tab=table&language=en&pcode=tps00001&tableSelection=1&footnotes=yes&labeling=labels&plugin=1

^18^Current and Historical Rate Tables. [cited 2015 Sept] Available from: http://www.xe.com/currencytables/?from=EUR&date=2008-01-01

^19^World Health Organization (WHO). Global policy report on the prevention and control of viral hepatitis IN WHO MEMBER STATES. 2013. [cited 2015 Aug] Available at URL: http://apps.who.int/iris/bitstream/10665/85397/1/9789241564632_eng.pdf?ua=1

^20^ECDC. Annual epidemiological report on communicable diseases in Europe 2009. [cited 2015 Sept] Available from: http://www.ecdc.europa.eu/en/publications/Publications/1011_SUR_Annual_Epidemiological_Report_on_Communicable_Diseases_in_Europe.pdf

^21^Cicchetti A. La tensión regulación- innovación en las decisiones de precio y re-embolso de nuevos medicamentos en Italia. [cited 2015 Jan] Available from: http://www.fgcasal.org/fgcasal/database/documentos/PharmaMar-FGC_2012_AMERICO_CICCHETTI-2.pdf

^22^HCV new drug research. Hepatitis C News; European Gastroenterologists Will Prescribe Telaprevir and Boceprevir to Nonresponder and Treatment-Naive Patients Following Launch [Internet]. 2011 Available from: http://hepatitiscnewdrugs.blogspot.dk/2011/04/hepatitis-c-news-european.html (Accessed 10 Oct 2015).

^23^Incivek set to break record for fastest product launch [Internet]. EvaluatePharma. [cited 2015 Nov]. Available from: http://epvantage.com/Universal/View.aspx?type=Story&id=261529&isEPVantage=yes

^24^Gilead Sciences Announces First Quarter 2014 Financial Results [Internet]. Gilead Sciences Inc. 2014. [cited 2015 Nov] Available from: http://www.gilead.com/news/press-releases/2014/4/gilead-sciences-announces-first-quarter-2014-financial-results [Internet] (Accessed 8 July 2016).

^25^PBAC. Australian Government Department of Health. March 2015 PBAC MEETING – POSITIVE RECOMMENDATIONS. [Cited Sept 2015]. Available from: http://www.pbs.gov.au/info/industry/listing/elements/pbac-meetings/pbac-outcomes/2015-03.

^26^Hepatitis C Society. Sofosbuvir Cost. Available from URL: http://esofosbuvir.com/sofosbuvir-drug/sofosbuvir-cost/ (Accessed 8 July 2016).

^27^PMlive. France agrees lowest Sovaldi pricing in EU. Government brings cost of hepatitis C drug to €5,000 below list price. Available at URL: http://www.pmlive.com/pharma_news/france_agrees_lowest_sovaldi_pricing_in_eu_618661 (Accessed 8 July 2016).

^28^Hepatitis News. French Strike Deal for Sofosbuvir. Available at URL: https://gareth-williams-gcuc.squarespace.com/hepatitis-articles/2015/10/26/french-strike-deal-for-sofosbuvir?rq=french-strike-deal-for-sofosbuvir (Accessed 8 July 2016).

^29^Avis relatif aux prix de spécialités pharmaceutiques publiés en application de l'article L. 162-16-5 du code de la sécurité sociale. Available at URL: https://www.legifrance.gouv.fr/affichTexte.do?cidTexte=JORFTEXT000030741836 (Accessed 8 July 2016).

^30^Irish Times. How to sell a $1000 pill for $10 without losing money. Available at URL: http://www.irishtimes.com/business/health-pharma/how-to-sell-a-1-000-pill-for-10-without-losing-money-1.2554351 (Accessed Oct 2015).

^31^Messori (2015b). Available from: http://www.bmj.com/content/351/bmj.h4988/rr (Accessed 8 July 2016).

^32^Daily Maverick. Health-e: South Africa's “other” virus. http://www.dailymaverick.co.za/article/2015-11-30-health-e-south-africas-other-virus/#.V3q1oqSzHIU (Accessed Feb 2016).

^33^Campillo-Artero, C. The merry-go-round of approval, pricing and reimbursement of new drugs (Part 2). Available at URL: http://www.hspm.org/countries/spain25062012/livinghit.aspx?Section=3.2%20Population%20coverage%20and%20basis%20for%20entitlement&Type=Section#6Themerry-go-roundofapproval,pricingandreimbursementofnewdrugs(Part2) (Accessed 8 July 2016).

^34^CNAMTS. Ameliorér la qualité du système de sante et maîtriser les depenses. Propositions de l'Assuarance Maladie pour 2016. [Internet]. Available from: http://www.ameli.fr/rapport-charges-et-produits-2016/ (Accessed Feb 2016).

^35^World Health Organization “19th WHO Model List of Essential Medicines (April 2015)”. Geneva. Available at URL: http://www.who.int/medicines/publications/essentialmedicines/EML2015_8-May-15.pdf (Accessed Oct 2015).
